The article "Artichoke Leaf Extract-Mediated Neuroprotection against Effects of Aflatoxin in Male Rats" was published in 2022. Journal: Biomed Res Int.

# Artichoke Leaf Extract-Mediated Neuroprotection against Effects of Aflatoxin in Male Rats

**DOI:** 10.1155/2022/4421828

**Published:** 2022-07-19

**Authors:** Enas A. Ibrahim, Mokhtar I. Yousef, Doaa A. Ghareeb, Maria Augustyniak, John P. Giesy, Mourad A. M. Aboul-soud, Abeer El Wakil

**Affiliations:** ^1^Department of Environmental Studies, Institute of Graduate Studies and Research, Alexandria University, Egypt; ^2^Bioscreening and Preclinical Trial Lab, Biochemistry Department, Faculty of Science, Alexandria University, Egypt; ^3^Biochemistry Department, Faculty of Science, Alexandria University, Egypt; ^4^Pharmaceutical and Fermentation Industries Development Centre, The City of Scientific Research and Technological Applications, Alexandria, Egypt; ^5^Institute of Biology, Biotechnology and Environmental Protection, Faculty of Natural Sciences, University of Silesia in Katowice, Bankowa 9, 40-007 Katowice, Poland; ^6^Department of Veterinary Biomedical Sciences & Toxicology Centre, University of Saskatchewan, Saskatoon, SK, Canada S7N5B3; ^7^Department of Integrative Biology, Michigan State University, East Lansing, MI 48895, USA; ^8^Department of Environmental Science, Baylor University, Waco, TX 76798-7266, USA; ^9^Chair of Medical and Molecular Genetics Research, Department of Clinical Laboratory Sciences, College of Applied Medical Sciences, King Saud University, P.O. Box 10219, Riyadh 11433, Saudi Arabia; ^10^Department of Biological and Geological Sciences, Faculty of Education, Alexandria University, Egypt

## Abstract

Attenuation of adverse effects of aflatoxin (AFB_1_) in brains of B_1_ rats by extracts of leaves of artichoke was studied. The active ingredients in extracts of leaves of artichoke, *Cynara scolymus* L., were determined by HPLC analysis. In the 42-day experiment, rats were exposed to either sterile water, 4% DMSO, 100 mg artichoke leaf extract/kg body mass, 72 *μ*g aflatoxin B_1_/kg body mass, or AFB_1_ plus artichoke leaf extract. Neurotoxicity of AFB_1_ was determined by an increase in profile of lipids, augmentation of plasmatic glucose and concentrations of insulin, oxidative stress, increased activities of cholinergic enzymes, and a decrease in activities of several antioxidant enzymes and pathological changes in brain tissue. Extracts of artichoke leaf significantly reduced adverse effects caused by AFB_1_, rescuing most of the parameters to values similar to unexposed controls, which demonstrated that adverse, neurotoxic effects caused by aflatoxin B_1_ could be significantly reduced by simultaneous dietary supplementation with artichoke leaf extract, which itself is not toxic.

## 1. Introduction

Mycotoxins are toxic fungal products that thrive in human food and animal feed, causing disease and death in humans and animals, when consumed in concentrations exceeding the limits [1, 2]. These toxigenic fungi contaminating agricultural grains have been divided into two groups. The first are those that invade seed crops and are known as “field” fungi and include species of the genera *Alternaria*, *Fusarium*, and *Cladosporium*, which reputedly gain access to seeds during plant development. The second class is described as “storage” fungi and includes species from the genera *Penicillium* and *Aspergillus* that proliferate during storage [3]. Both *Aspergillus flavus* and *Aspergillus parasiticus* produce aflatoxins (AFs) that can infect crops before harvesting. Contamination of field crops with aflatoxins causes losses of agricultural commodities in many zones of the world [4]. Therefore, it is necessary to control AF contamination in food and feed to ensure food safety and, more importantly, to safeguard human and animal health.

The article "Artichoke Leaf Extract-Mediated Neuroprotection against Effects of Aflatoxin in Male Rats" was published in 2022. Journal: Biomed Res Int.

Aflatoxin B1 (AFB_1_) is considered the most significant risk factor among mycotoxins and the most frequently found aflatoxin in contaminated foods and feed [5–7]. Due to its stability and heat-resistant nature, not all food processing methods are efficient at removing AFB_1_. Therefore, public health can be affected following dietary exposure to AFB_1_. On a worldwide basis, the safe limits of aflatoxin B_1_ range from 4 to less than 30 *μ*g/kg for human consumption [8]. AFB_1_ may increase lipid peroxidation, which contributes to cytotoxic damage in many organs, especially the brain, leading to neurodegenerative diseases and weakening of this organ's function [9, 10]. Furthermore, it has been documented that prenatal administration of AFB_1_ in rat offspring can delay development of reflex responses, learning ability, motor activity, locomotor coordination, and exploratory behavior [11]. It can also cause tumors in both the central and peripheral nervous systems and various nonepithelial neurogenic tumors. In the central nervous system, neurons have a high metabolic rate and a low capacity for anaerobic metabolism. As a result, when the oxygen supply to the brain is insufficient, the neuronal brain cells degenerate within minutes. AFB_1_ has been reported to alter concentrations of neurotransmitters in brains of rats [12]. While drug-based chemoprotection strategies can be useful in mitigating toxicity of aflatoxins, due to the large numbers of persons potentially affected, practical implementation is limited. Therefore, it is imperative to identify alternative treatments where patients could benefit from fewer complications and a better quality of life. In recent years, renewed interest in natural products has spotlighted drug discovery and cancer research [13, 14]. In the present study, an approach to counteract neurotoxicity caused by AFB_1_ was investigated in which diets were supplemented with an entirely natural, plant-based product, extracts of leaves of artichoke. The alternative therapy if effective would be cost-effective and result in fewer side effects.

The article "Artichoke Leaf Extract-Mediated Neuroprotection against Effects of Aflatoxin in Male Rats" was published in 2022. Journal: Biomed Res Int.

The artichoke, *Cynara scolymus L.*, is a member of the *Asteraceae* family and a native plant of the Mediterranean. Because of its nutritional benefits and medicinal properties, *C. scolymus L.* is cultivated worldwide. Officially, medicinal artichoke products consist of dried leaves. It is a rich source of polyphenolic compounds, mainly caffeoylquinic acids, and flavonoids, isolated from the plant polar extracts, together with the polysaccharide inulin, fibers, and minerals. The lipophilic fraction comprises fatty acids, triterpenes, and sesquiterpenes as major metabolites [15]. Using the International Union of Pure and Applied Chemistry (IUPAC) nomenclature, the plant contains up to 6% phenolic acids, including 5-O-caffeoylquinic acid (chlorogenic acid), which is the most abundant substance (39%), followed by 1,5-O-dicaffeoylquinic acid (21%) and 3,4-O-dicaffeoylquinic acid (11%), based on total caffeoylquinic acid content. The artichoke also contains up to 5% sesquiterpene lactones, with cynaropicrin being the primary component. Other ingredients are dehydrocynaropicrin, grosheimin and their derivatives, and 0.35-0.75% flavonoids, including scolymoside, cynaroside, and cyanotrioside [16]. Furthermore, the 1,3-O-dicaffeoylquinic acid (cynarin) content in methanolic extracts of the artichoke is small, about 1.5%, the majority of which is located in the pulp of the leaves, although the dried leaves and stems of artichoke also contain this compound [15].

Phenolic substances contained in artichoke have an essential scavenging activity against reactive oxygen species (ROS) and free radicals and perform as a protective shield against oxidative damage to biological molecules, such as proteins, lipids, and DNA [17]. Gebhardt [18] reported that 1,3-dicaffeoylquinic acid and flavonoids were considered choleretic, anticholestatic, and diuretic, reducing cholesterol. While the plant and its preparations are commonly used to treat dyspepsia, they are also used traditionally to prevent and treat atherosclerosis and kidney dysfunction (diuretic) [19].

Effects of artichoke leaf extract (ALE) after 42 days of exposure in male rats were investigated. General pathological characteristics and specific brain plasma markers were evaluated. Besides, lipid profile, antioxidant enzyme activities, and free radicals were analyzed in the brain to elucidate the potential neuroprotective effects of ALE. Furthermore, the histopathological architecture of the brain was evaluated. In this study, the following hypothesis was tested: adverse neurotoxic effects caused by aflatoxin B_1_ can be significantly reduced by simultaneous dietary supplementation with extracts of leaves of artichoke.

The article "Artichoke Leaf Extract-Mediated Neuroprotection against Effects of Aflatoxin in Male Rats" was published in 2022. Journal: Biomed Res Int.

## 2. Materials and Methods

### 2.1. Chemicals

AflatoxinB_1_ powder (C_17_H_12_O_6_) from *Aspergillus flavus* was purchased from Sigma-Aldrich, France (CAS Number 1162-65-8, Product Number A6636-10MG, purity 99.7% and formula mass: 312.27). Commercial ALE (super artichoke, capsules) was produced by Western Pharmaceutical Industries, Cairo, Egypt, and used in this study. All reagents and chemicals were of analytical grade.

### 2.2. Animals

Twenty-five 12-week-old male albino rats were used for this research. The rats were obtained from the Medical Research Institute (Center of Medical Technology), Alexandria University, Egypt. They were housed in clean cages with hardwood bedding. They had access to feed and clean tap water *ad libitum*. Animals were maintained in a controlled atmosphere at a temperature of 25 ± 5°C and 50-70% humidity, and they were subjected to standard 12 h light and dark cycles.

### 2.3. The Active Ingredient of the Artichoke, Cynara scolymus L., Leaf Extract

HPLC analysis was carried out using an Agilent 1260 series. Separations were conducted by use of an Eclipse C18 column (4.6 mm × 250 mm, 5 *μ*m). Water and 0.05% trifluoroacetic acid in acetonitrile were used at a flow rate 1 mL/min as mobile phases A and B, respectively. The gradient was programmed consecutively in a linear manner as follows: 0 min (82% A), 0–5 min (80% A), 5-8 min (60% A), 8-12 min (60% A), 12-15 min (82% A), 15-16 min (82% A), and 16-20 (82% A). The multiwavelength detector was monitored at 280 nm. The injection volume was 5 *μ*L for each of the sample solutions. The column temperature was maintained at 40°C.

### 2.4. Treatment Protocol

Rats were allowed to acclimatize to their environment for two weeks before the experiment started. They were randomly divided into five treatment groups of five rats each and treated with sterile water, control group; 4% DMSO (1 mL/kg body mass), which is the solvent for AFB_1_, DMSO group; ALE (100 mg/kg, bm), ALE group; AFB_1_ at the concentration of 72 *μ*g/kg, bm (as 1/100 of LD50% dose: 7.2 mg/kg, bm), AFB1 group; and AFB_1_ plus ALE, ALE+AFB1 group. Animals were orally gavaged daily with the respective doses for 42 consecutive days. The initial and final body masses of male rats were recorded in each treatment group, and they did not show any significant change among the treated groups.

The article "Artichoke Leaf Extract-Mediated Neuroprotection against Effects of Aflatoxin in Male Rats" was published in 2022. Journal: Biomed Res Int.

### 2.5. Blood and Brain Collection

Animals were euthanized at the end of the experimental period, by use of isoflurane (2 mL/kg, bm) by inhalation. Blood was collected by cardiac puncture in test tubes containing heparin. Plasma was obtained from whole blood by centrifugation at 860 × *g* for 20 min. Blood plasma was kept at −80°C until analysis. Brains were removed, released from adhering fat and connective tissues, washed with chilled saline solution (0.9%), dried on tissue paper, and mass determined. A portion of the brain was immediately kept in 10% formalin for histological studies. Another portion of 2 g of the brain was minced and homogenized (10%, *w*/*v*), separately, in ice-cold phosphate buffer (0.25 M, pH 7.4) in a Potter–Elvehjem type homogenizer. Homogenates were centrifuged at 10,000 × *g* for 20 min at 4°C to pellet cell debris, and the supernatant was collected and stored at −80°C for further analyses.

### 2.6. Biochemical Analysis

The tests were performed using a UV-visible spectrophotometer.

#### 2.6.1. Plasma Lipid Profile

The plasma lipid profile was performed by measuring concentrations of total lipid (Cat. No. TL20 10), cholesterol (Cat. No. CH12 20), triglycerides (Cat. No. TR20 30), high-density lipoprotein (HDL) (Cat. No. CH12 30), and low-density lipoprotein (LDL) (Cat. No. CH12 31). Analyses were done by colorimetric methods using commercial kits (BioDiagnostic Inc., Cairo, Egypt). Concentrations of VLDL in blood plasma were calculated according to Friedewald's equation [20].

#### 2.6.2. Estimation of Plasma Glucose, Insulin Concentration, and Homeostasis Model Assessment (HOMA)

Concentrations of glucose were quantified by use of a colorimetric method using a commercially available kit (Cat. No. GL13 20, BioDiagnostic Inc., Cairo, Egypt). Concentrations of insulin were measured by ELISA with the assay kit according to the manufacturer's instructions (Bioneovan Ltd., Beijing, China). The homeostasis model assessment of insulin resistance (HOMA-IR) index and the function of the pancreatic *β*-cells (HOMA-B) provided valid and reliable information based on the fasting plasma glucose level and insulin concentration. HOMA-IR and HOMA-B were calculated with a formula adapted by Matthews et al. [21].

#### 2.6.3. TNF-*α*, IDO, and TIMP3 Assays

ELISAs were performed for these parameters as per the manufacturer's instructions. The ELISA kits for tumor necrosis factor-alpha (TNF-*α*), indoleamine-pyrrole 2,3-dioxygenase (IDO), and tissue inhibitor metallopeptidase (TIMP3) were obtained from Bioneovan Ltd., Beijing, China.

The article "Artichoke Leaf Extract-Mediated Neuroprotection against Effects of Aflatoxin in Male Rats" was published in 2022. Journal: Biomed Res Int.

#### 2.6.4. Brain Free Radicals and Antioxidant Enzyme Assays

Concentrations of thiobarbituric acid reactive substances (TBARS) (Ref. MD25 29), uric acid (UA) (Ref. UR21 20), and nitric oxide (NO) (Ref. NO25 33) and the activity of superoxide dismutase (SOD) (Ref. SD25 21), glutathione S-transferase (GST) (Ref. GT25 19), and glutathione peroxidase (GPx) (Ref. GP25 24) in brain supernatants were determined spectrophotometrically by use of commercially available assay kits obtained from the BioDiagnostic Company (Cairo, Egypt). Measurements of the above parameters were performed strictly according to the manufacturer's instructions. Urea was measured in the plasma by the urease-Berthelot method [22] (Ref. UR21 20, BioDiagnostic Inc., Cairo, Egypt). Glutathione level (GSH) was determined following the method of Jollow et al. [23], and xanthine oxidase (XO) activity was measured according to Litwack et al. [24].

#### 2.6.5. Estimation of the Activities of Acetylcholinesterase (AChE) and Monoamine Oxidase (MAO)

AChE activity was estimated according to Ellman's method [25]. It was measured spectrophotometrically at 405 nm and expressed as *μ*mol/min/mg protein. MOA activity was determined as described by Hallman et al. [26], where 1 mL of 50 mM sodium phosphate buffer pH 7.4, 150 *μ*L brain supernatant, and 500 *μ*L of 5 mM benzylamine were mixed well. MAO activity (U/l) = ∆A × total volume × 1000/3.2 × brain supernatant volume. The absorbance was measured at 250 nm against air after 30 s and 90 s.

### 2.7. Histopathology

The brain sections were assessed histologically, using the H&E staining method, to provide general knowledge concerning the potential aflatoxin B_1_ influence on tissue structure compared to the control and ALE treatment alone. Combined treatment using AFB_1_ and ALE (ALE+AFB1 group) has also been assessed to evaluate the potential beneficial effects of ALE on the brain. Brain tissues, fixed in 10% formalin immediately after collecting, were processed by cutting pieces in tissue cassettes with an automated tissue processor. They were then embedded in paraffin and, after that, were sectioned with microtome at 4-6 mm thickness. Slides were then stained with hematoxylin and counterstained with eosin for histological examination. Photographs were taken on an Olympus XC30 microscope (Germany) with a digital camera (Olympus UC30 camera). Representative pictures were taken at 20x and 40x magnification from each group.

### 2.8. Statistical Analysis

Statistical analysis was performed using Statistica 13.1. All biochemical measurements were performed in 5 replicates. The distribution of the data (the Kolmogorov-Smirnov and Shapiro-Wilk tests) and homogeneity of variance (the Levene test) was checked before analysis. The data fulfilled analysis of variance criteria; therefore, parametric tests were used: ANOVA (post hoc LSD test, *p* < 0.05), and the differences between experimental groups were investigated. All parameters were expressed as the mean ± SD in the figures. Principal component analysis (PCA) was also performed for all measured parameters.

The article "Artichoke Leaf Extract-Mediated Neuroprotection against Effects of Aflatoxin in Male Rats" was published in 2022. Journal: Biomed Res Int.

## 3. Results and Discussion

### 3.1. Chemical Composition of the Artichoke Leaf Extract

The analysis of artichoke capsule identified 17 components (Figure 1). Apart from some components, such as pyrocatechol, ferulic acid, naringenin, catechin, and gallic acid, the artichoke's highest component concentration was the chlorogenic acid (CGA). CGA has been found to have anti-inflammatory, antioxidant, antiviral, antibacterial, lipid lowering, hypoglycemic, and cardioprotective properties and many other pharmacological benefits [27]. Therefore, CGA may play an important role in health promotion.

### 3.2. Plasma Lipid Profile

Treatment of the rats with ALE for 42 days resulted in a significant (*p* ≤ 0.05) decrease in total plasma lipids (412.0 ± 12.2 mg/dL), cholesterol (105.3 ± 1.8 mg/dL), triglycerides (139.4 ± 5.8 mg/dL), low-density lipoprotein (LDL; 33.1 ± 12.2 mg/dL), and very-low-density lipoprotein (VLDL; 27.9 ± 1.2 mg/dL) compared to control (562.6 ± 25.9, 160.3 ± 16.9, 152.6 ± 6.5, 96.1 ± 11.9, and 30.5 ± 11.9 mg/dL, respectively). Simultaneously, a significant (*p* ≤ 0.05) increase in the concentration of high-density lipoproteins (HDL: 44.4 ± 2.9 mg/dL vs. control: 33.8 ± 3.2 mg/dL) in the plasma of rats from the ALE group was found (Figure 2). Compared to all other groups, aflatoxin B_1_ caused a significant increase in almost all lipid profiles' parameters (total lipids: 705.2 ± 16.3 mg/dL; cholesterol: 211.9 ± 17.2 mg/dL; triglycerides: 173.0 ± 10.2 mg/dL; LDL: 146.1 ± 10.3 mg/dL; and VLDL: 34.6 ± 2.0 mg/dL). The only exception was found for HDL (25.6 ± 2.1 mg/dL), where a significant decrease in concentration in the AFB1 group was noted compared to the rest of the experimental groups (Figure 2(d)). The administration of ALE combined with aflatoxin B_1_ (ALE+AFB1 group) reduced the concentration of total lipids (537.0 ± 12.6 mg/dL), cholesterol (164.9 ± 12.8 mg/dL), HDL (34.4 ± 2.7 mg/dL), and LDL (107.5 ± 10.7 mg/dL) to the values typical for the control group (Figures 2(a) and 2(b) and 2(d) and 2(e)). Moreover, both factors' combined use resulted in a significant reduction in triglycerides (116.4 ± 13.9 mg/dL) and VLDL (23.3 ± 2.8 mg/dL) concentration compared to the control group (Figures 2(c) and 2(f)).

When studying the brain, lipids are of particular interest because they account for more than 50% of its dry mass. They are the main components of cell membranes and are repositories of chemical energy. The crucial role of lipids in brain physiology and cell signaling has been demonstrated by neurologic disorders and several neurodegenerative diseases in which lipid metabolism is altered [28]. Previously, lipid content of the brain was considered relatively resistant to change induced by dietary intake [29, 30]. However, results presented here show that ALE consumed simultaneously with aflatoxin B_1_ for 42 days downregulated almost all lipid profile parameters except HDL, which was upregulated following exposure to AFB_1_ alone. In brief, it is evident that ALE could positively alter lipid content and function of the rat brain. The positive effect of ALE is undoubtedly related to the interaction of the active ingredients of the extract, mainly chlorogenic acid. It is known that some derivatives of CGA may affect lipid metabolism significantly by decreasing the oxidation of low-density lipoproteins (LDL) and total cholesterol. A reduction of cholesterol and triacylglycerols concentrations by 44% and 58% was observed in obese, hyperlipidemic, and insulin-resistant Zucker rats, infused with CGA at a dose of 5 mg/kg body weight/day for three weeks [31]. One of the first hypotheses explaining the action of CGA was that of its cations' chelation properties resulting in oxidative stress inhibition [32]. More recent studies show that this compound can lower cholesterol and positively affect lipid metabolism by upregulating gene expression of a peroxisome proliferation-activated receptor (PPAR-*α*). This nuclear receptor acts as a transcription factor regulating the expression of genes related to metabolism including lipid metabolism [33]. Our research shows that ALE, containing CGA as its main component, improves lipid metabolism when disrupted by AFB1.

The article "Artichoke Leaf Extract-Mediated Neuroprotection against Effects of Aflatoxin in Male Rats" was published in 2022. Journal: Biomed Res Int.

### 3.3. Plasma Glucose and Insulin Concentration, HOMA-IR, and HOMA-B Index

Exposure to ALE or AFB_1_ alone resulted in different responses. Treatment with ALE alone caused no significant effect on insulin concentration (4.4 ± 0.2 *μ*U/mL) and the homeostatic model assessment for insulin resistance (HOMA-IR; 0.9 ± 0.04) index, but the concentration of glucose (84.2 ± 1.0 mg/dL) was slightly less, and the homeostatic model assessment for beta cells (HOMA-B; 18.7 ± 0.04) index was elevated compared to the control group (4.3 ± 0.2, 1.0 ± 0.1, 91.4 ± 8.1, and 16.8 ± 1.5, respectively) (Figure 3). Aflatoxin B_1_ resulted in significantly greater concentrations of glucose (116.4 ± 4.8 mg/dL) and insulin (4.8 ± 0.1 *μ*U/mL) in blood plasma of rats and the HOMA-IR index (1.38 ± 0.1) compared to rats in all other groups. Furthermore, in rats exposed to AFB1, the HOMA-B index (14.9 ± 0.8) was significantly less than in the other groups. The treatment of AFB1-exposed rats with ALE restored the levels of glucose (97.6 ± 5.6 mg/dL), insulin (4.2 ± 0.2 *μ*U/mL) and HOMA (HOMA-IR: 1.0 ± 0.1 and HOMA-B: 15.7 ± 1.1) indices.

Insulin is pivotal for maintaining glucose metabolism in the periphery and the brain [34]. Alterations in the insulin regulation system lead to hyperinsulinemia, which produces widespread insulin resistance. The latter is a state in which tissues that require glucose have a diminished response to insulin, and the subsequently reduced clearance of glucose from the blood feeds back onto the pancreas to increase secretion of insulin to induce glucose uptake [35]. Results of the current study confirmed previous findings where exposure to AFB_1_ increased insulin resistance, as shown by the decrease in HOMA-B values associated with elevated HOMA-IR values, which corresponds to decreased insulin effectiveness in regulating plasma glucose. However, simultaneous exposure to ALE and AFB_1_ positively affects the discussed parameters and brings them to the control level.

The positive effect of artichoke extract can be again associated with the impact of chlorogenic acid. Mentioned above studies by Rodriguez de Sotillo and Hadley [31] on Zucker rats also showed that CGA did not promote sustained hypoglycemia and improved glucose tolerance. Underlying mechanisms include the influence of CGA on the glucose-6-phosphatase activity involved in glucose metabolism [36]. Also, an improved insulin sensitivity after CGA treatment can increase glucose uptake by tissues. It has been shown that phenolic acids improve insulin sensitivity of HepG2 cells by reducing the insulin signaling blockade and modulation of glucose consumption [37]. Therefore, a decrease in insulin and glucose concentrations is connected with decreased synthesis of lipids [31].

### 3.4. TNF*α*, IDO, and TIMP3 in the Brain of Rats

Treatment of rats with ALE had no significant influence on concentrations of tumor necrosis factors *α* (TNF*α*; 1302.0 ± 25.5 pg/mg protein), indoleamine-pyrrole 2,3-dioxygenase (IDO; 1563.8 ± 56.4 pg/mg protein), and tissue inhibitor metallopeptidase (TIMP3; 4027.5 ± 259.5 pg/mg protein) (Figure 4). Aflatoxin B_1_ administered alone for 42 days caused a significant (*p* < 0.05) increase in TNF*α* (2387.5 ± 31.8 pg/mg protein) and IDO (2334.5 ± 129.4 pg/mg protein) and, at the same time, a decrease in concentrations of TIMP3 (773.0 ± 45.2 pg/mg protein) compared to controls (1298.5 ± 2.1, 1542.7 ± 41.9, and 3821.0 ± 74.9 pg/mg protein, respectively). These evaluated parameters were generally positively influenced by the administration of AFB_1_ together with ALE (ALE+AFB1 group). The concentration of TNF*α* value (1658.5 ± 30.4 pg/mg protein) in rats exposed to ALE+AFB1 was less than that found in the rats exposed to AF1 alone but was still greater than in the control group. The mean IDO value (1726.0 ± 74.7 pg/mg protein) in brains of rats exposed to ALE+AFB1 was similar to that of the control group (1542.7 ± 41.9 pg/mg protein). Concentrations of TIMP3 (2274.0 ± 142.8 pg/mg protein) in brains of rats exposed to AFB_1_ and ALE simultaneously were greater than in those exposed to AFB_1_ alone (779.0 ± 45.2 pg/mg protein), but still significantly less compared to unexposed rats in the control group (3821.0 ± 74.9 pg/mg protein).

The article "Artichoke Leaf Extract-Mediated Neuroprotection against Effects of Aflatoxin in Male Rats" was published in 2022. Journal: Biomed Res Int.

TNF-*α* is a proinflammatory cytokine that is upregulated in response to various injuries in the hippocampi of the ischemic brain [38] and chronically stressed rats [39]. Consistent with results of previous studies, exposure to AFB_1_ in the present study affects the concentrations of various inflammatory markers in brains of rats, including proinflammatory cytokines (TNF-*α*) and tissue inhibitor of metalloproteinases (TIMP3). Results of previous studies have provided evidence that TNF can protect neurons by encouraging the expression of antiapoptotic and antioxidative proteins [40]. Furthermore, experiments with TNF-deficient mice indicate that although TNF has a deleterious effect during the acute response in a traumatized brain, it also plays a crucial part in both the long-term behavioral recovery and the histological repair of the tissues. Alterations of the IDO pathway have also been reported in several neurological diseases, including stroke, multiple sclerosis, Parkinson, Alzheimer, and schizophrenia [41], similar to our experiment. It has been documented that TIMP3 is involved in regulating cellular processes, such as cell proliferation, apoptosis, and angiogenesis [42]. Combined exposure to ALE and aflatoxin B_1_ (ALE+AFB1) confirmed the beneficial effect of ALE on these parameters by alleviating the toxic damage caused by AFB_1_ alone and restoring their normal values.

Phenolic acids, also CGA, can reduce tissue inflammation and apoptosis of nerve cells and stimulate brain cell protection [43]. The latest research by Shah et al. [44] showed that CGA could counteract oxidative stress in the ischemic cerebral cortex, lower proinflammatory protein expression, and reduce histopathological changes. The anti-inflammatory effect of CGA was related to the regulation of nuclear factor kappa B (NF-*κ*B), IL-1*β*, and TNF-*α*. Our research shows that artichoke extract, rich in phenolic acids, has neuroprotective effects through its influence on pro-inflammatory proteins.

The article "Artichoke Leaf Extract-Mediated Neuroprotection against Effects of Aflatoxin in Male Rats" was published in 2022. Journal: Biomed Res Int.

### 3.5. Oxidative Stress Level and Antioxidant Enzyme Activity

While aflatoxin B_1_ led to threefold increase in concentration of TBARS (34.8 ± 2.34 nmol/mg protein), ALE caused a significant reduction of this parameter (8.84 ± 0.88 pg/mg protein) in brains of rats compared to control (11.8 ± 0.8 pg/mg protein) (Figure 5(a)). Exposure to a combination of AFB_1_ and ALE (ALE+AFB1) reduced concentrations of TBARS (16.7 ± 1.4 pg/mg protein), compared to the aflatoxin B_1_-treated group (34.8 ± 2.34 pg/mg protein). However, the concentration remained greater than in the control group. The xanthine oxidase (XO) activity and concentration of uric acid (UA) were consistent with the TBRAS pattern and were significantly greater in rats exposed to AFB1 (XO: 67.9 ± 2.7 *μ*mol/h/mg protein and UA: 4.7 ± 0.4 mg/mg protein), compared to controls (XO: 39.5 ± 2.9*μ*mol/h/mg protein and UA: 2.3 ± 0.3 mg/mg protein) and all other groups (Figures 4(b) and 4(c)). The treatment of rats by AFB1 and ALE resulted in a reduction of XO activity (40.1 ± 4.1 *μ*mol/h/mg protein) and UA concentration (2.9 ± 0.3 mg/mg protein) compared to the rats from the AFB1 group (XO: 67.9 ± 2.7 *μ*mol/h/mg protein and UA: 4.7 ± 0.4 mg/mg protein).

Exposure of rats to ALE alone caused a significantly greater concentrations of glutathione (GSH: 4.9 ± 0.1 vs. control: 3.9 ± 0.1 *μ*mol/mg protein) and activities of superoxide dismutase (SOD: 11.6 ± 0.8 vs. control: 9.0 ± 0.7 nmol/min/mg protein), glutathione S-transferase (GST: 0.8 ± 0.04 vs. control: 0.6 ± 0.04 nmol/min/mg protein), and glutathione peroxidase (GPx: 0.21 ± 0.006 vs. control: 0.17 ± 0.02 U/mg protein). Aflatoxin B_1_ had the opposite effect on these parameters. After 42 days of exposure to AFB_1_, there was significantly less concentration of GSH (2.8 ± 0.2 *μ*mol/mg protein) and lesser activities of SOD (5.7 ± 0.7 nmol/min/mg protein), GST (0.4 ± 0.02 nmol/min/mg protein), and GPx (0.1 ± 0.02 U/mg protein), compared to all other groups. In rats exposed to AFB_1_ and ALE simultaneously, the concentration of GSH (3.5 ± 0.3 *μ*mol/mg protein) and activities of SOD (8.8 ± 0.6 nmol/min/mg protein), GST (0.6 ± 0.1 nmol/min/mg protein), and GPx (0.16 ± 0.02 U/mg protein) did not differ from values of unexposed rats (GSH: 3.9 ± 0.1 *μ*mol/mg protein; SOD: 9.0 ± 0.7 nmol/min/mg protein; GST: 0.6 ± 0.04 nmol/min/mg protein; and GPx: 0.17 ± 0.02 U/mg protein, respectively) (Figure 6). Consistent with the result of the present study, Surai [45] reported that AFB_1_ induced damage at both the cellular and tissue levels via the production of free radicals and lipid peroxides. Furthermore, Antonyak and Koval [46] revealed that SOD activity decreased compared to control values following AFB_1_ administration, while TBARS increased significantly in brain homogenates of experimental animals' group.

The article "Artichoke Leaf Extract-Mediated Neuroprotection against Effects of Aflatoxin in Male Rats" was published in 2022. Journal: Biomed Res Int.

Results of the present study were also consistent with those of previous studies that found that treatment with AFB_1_ leads to increased oxidative stress markers, including TBARS and decreased activities of different antioxidant enzymes, including GSH, SOD, GST, and GPx [47]. Also, oxidative stress catalyzes both hypoxanthine's conversion to xanthine and, in turn, to uric acid [48]. Uric acid is a potent plasma antioxidant that scavenges singlet oxygen, peroxy radicals, and hydroxyl radicals and has been studied extensively in many physiological and pathological systems, including neurodegenerative diseases [49]. Consistent with findings of the study, results of which are reported here, previous studies have found exposure to AFB_1_ caused harmful effects that cause depletion of the antioxidant defense system leading to oxidative stress and a reduction of amounts of GSH and activities of SOD and GST [50, 51]. Also, AFB_1_ exposure caused an obvious rise in XO levels.

In this study, exposure to ALE alone antioxidant content TBARS and XO levels was less than those in the control, but exposure to AFB_1_ resulted in lesser activities of variable antioxidant enzymes in rats. Simultaneous use of ALE together with AFB_1_ brings the levels of these parameters to control ones. This result is consistent with previous studies revealing that antioxidants may protect tissue from damage by adjusting the detoxification and promoting antioxidant systems [52, 53]. Other studies have shown that phenolic compounds, including CGA, exhibit neuroprotective effects by enhancing the antioxidant defense. This was the case with aluminum-induced [54] or arsenite-induced neurotoxicity in mice [55]. In the experiments, CGA supplementation led to a reduction in the neurotoxicity of the mentioned xenobiotics, which was manifested by an increase in activity of SOD, CAT, GPx, GST, GR, and AChE [54, 55]. In our study, the protective effect of ALE against AFB1 is also due to the enhancement of antioxidative defense, which finally contributes to the neuroprotective effect.

### 3.6. Acetylcholinesterase and Monoamine Oxidase Activity and Nitric Oxide and Concentrations of Urea

Administration of ALE to rats did not affect acetylcholinesterase (AChE: 7.6 ± 0.6 vs. control: 7.2 ± 0.5 *μ*mol/min/mg protein) and monoamine oxidase (MAO: 11470.0 ± 983.3 vs. control: 11049.1 ± 781.3 U/mg protein) activity. At the same time, aflatoxin B_1_ caused a significant increase in the activity of both enzymes (AChE: 14.5 ± 2.1 *μ*mol/min/mg protein and MAO: 16435.8 ± 683.6 U/mg protein). AChE (9.4 ± 0.8 *μ*mol/min/mg protein) and MAO (12890.8 ± 1578.8 U/mg protein) activity in the rats from the ALE+AFB1 group was significantly lower than those in rats exposed to ABF1 alone (AChE: 14.5 ± 2.1 *μ*mol/min/mg protein and MAO: 16435.8 ± 683.6 U/mg protein), but still greater than that of the control group (AChE : 7.2 ± 0.5 *μ*mol/min/mg protein and MAO: 11049.1 ± 781.3 U/mg protein) (Figures 7(a) and 7(b)). ALE significantly increased nitric oxide concentration (NO: 6.5 ± 1.0 vs. control: 4.9 ± 0.3 nmol/mg protein) in brains of rats, while exposure to AFB_1_ alone (4.6 ± 0.8 nmol/mg protein) did not affect this parameter. Exposure to both factors simultaneously (ALE+AFB1) caused a significant increase in concentrations of NO (6.0 ± 0.3 nmol/mg protein), compared to the control group (4.9 ± 0.3 nmol/mg protein) (Figure 7(c)). Neither exposure to AFB1 alone nor ALE had significant had significant effects on concentrations of urea in brains of rat (control: 8.7 ± 1.6; ALE: 8.6 ± 2.0; AFB1: 8.1 ± 1.1; and ALE+AFB1: 9.6 ± 1.1 mg/dL) (Figure 7(d)).

The article "Artichoke Leaf Extract-Mediated Neuroprotection against Effects of Aflatoxin in Male Rats" was published in 2022. Journal: Biomed Res Int.

Cholinergic dysfunction is a prime sign of neurotoxicity. Herein, the toxicity of AFB_1_ in the brain was characterized by a significant increase in AChE activity, which is in agreement with results of previous studies [56]. Such increase in AChE activity due to exposure to AFB_1_ can be attributed to increased production of ROS that has been found to enhance the peroxidation of the plasma membrane, thereby affecting the integrity and functionality of the cholinergic system [57]. Exposure of rats to AFB_1_ significantly enhanced activity of MAO in the brain. MAO was previously shown to augment oxidative stress [58]. Simultaneous exposure to ALE and AFB_1_ in the present study supports the normalization of both enzyme activity to values close to the control group. The ameliorative effect of ALE may be attributed mainly to its antioxidant action and its ability to scavenge free radicals.

### 3.7. Relationships among Parameters

To estimate the relationship among all studied parameters, a PCA analysis was performed for all of them together (Figure 8) where the principal component 1 (PC 1) explained nearly 70% of the total variability. PC 1 was strongly created by GSH, HDL, GST, GPx, SOD, and TIMP3 (PC 1 positive values). However, for LDL, MAO, glucose, cholesterol, total lipids, UA, XO, TBARS, HOMA-IR, TNF*α*, and IDO1, negative PC values 1 were obtained. AChE, insulin, VLDL, and triglycerides had less effect on PC 1, while NO and urea were only weakly related to it. PC2 explained a little more than 10% of the overall variability in the data. Overall, the developed PCA model (PC1+PC2) explained approximately 80% of all parameters' variability (Figure 8(a)).

The article "Artichoke Leaf Extract-Mediated Neuroprotection against Effects of Aflatoxin in Male Rats" was published in 2022. Journal: Biomed Res Int.

A case-based PCA analysis identified three clusters (Figure 8(b)). The first cluster was created by data obtained from aflatoxin B_1_-treated rats. The second cluster, located on the opposite side of the scale and visibly separated from the others, included data from the group treated with ALE. The third cluster, however, quite scattered in the 2D plot space, was made up of data from control, DMSO, and ALE+AFB1 groups. There was no clear division between these three groups.

Results of the PCA analysis confirm that exposure of rats to AFB_1_ significantly influences the parameters discussed. The use of ALE also has a significant effect on animals, and this effect is opposite to that caused by aflatoxin. It can be assumed that the organism's functions are improved in AFB1+ALE-treated rats that showed reestablishment of almost all studied parameters. The combined exposure to AFB_1_ and ALE caused a return to a state similar to the control group.

### 3.8. Brain Histology

The brain sections were assessed histologically using the hematoxylin and eosin (H&E) staining method to determine the effects of AFB_1_, ALE alone, and in combination. Representative pictures were taken at 4x, 20x, and 40x magnification from each treated group. The assessment focused on the histopathological changes in the hippocampus and its corresponding dentate gyrus (DG). The hippocampus consists of the twisted dentate gyrus with an open concave part directed to the hippocampus. The hippocampus is divided into three subfields: cornu ammonis 1 (CA1), cornu ammonis 2 (CA2), and cornu ammonis 3 (CA3) (Figure 8 – control group). The CA1 region of the hippocampus consists of three layers: stratum pyramidalis (Sp), stratum radiatum (Sr), and stratum oriens (So). The primary cell type of striatum pyramidalis is composed of pyramidal cells that are characterized by well-demarcated rounded nuclei and prominent nucleoli (Figure 9 – control group). Unexposed rats and those exposed to ALE histological structures of the hippocampus and dentate gyrus were similar and determined to be normal, while the group treated with AFB_1_ exhibited cellular disorganization and degeneration manifested by darkly stained nuclei and extensive vacuolations with pyknotic hyperchromatic eccentric nuclei (Figure 9 – AFB_1_ group). Significantly, the treatment of AFB1-exposed rats with artichoke extract relieved these pathological changes (Figure 9 – ALE+AFB_1_ group).

The article "Artichoke Leaf Extract-Mediated Neuroprotection against Effects of Aflatoxin in Male Rats" was published in 2022. Journal: Biomed Res Int.

Histopathological assessment of the dentate gyrus in rats exposed to AFB_1_ exhibited a decrease in the dentate gyrus's granule cell layer thickness compared to the control group. Such a decrease in thickness of the dentate gyrus's main layer results mainly from the degenerative changes of nerve cells in this area. Moreover, glial proliferation, where microglia cells' infiltration was observed, was well manifested in the sections after exposure to AFB_1_ exposure. The ALE+AFB_1_ group revealed an improvement compared to the group treated with Aflatoxin B1 alone.

Herein, the AFB_1_-induced neurotoxicity as manifested by free radicals' augmentation, cholinergic enzymes, lipid profile, TNF-*α*, and IDO, finds its confirmation in histopathological architecture. Degenerative changes in the hippocampus's pyramid cells and nerve cells in the dentate gyrus were observed. Moreover, inflammatory infiltrations of microglia cells and macrophages were reported. Simultaneous use of ALE with AFB_1_ (ALE+AFB_1_ group) attenuates almost all histopathological alterations induced by a single exposure to AFB_1_. Results of previous studies are consistent with the results observed in this study [59–61].

To sum up, differential concentration of a variety of phenolic compounds has been reported in the artichoke leaf extract capsule in this study. CGA, which is the highly concentrated component in the extract, has been found previously to have several pharmacological properties including antioxidant, anti-inflammatory, lipid lowering, hypoglycemic, antibacterial, antiviral, cardioprotective, anticancer, and immunomodulatory. Therefore, the attenuation of the adverse effects of AFB1 as well as health promotion could be attributable to the phenolic composition of the artichoke leaf extract.

## 4. Conclusions

Results of the study presented here demonstrate adverse effects of AFB_1_ on brain function. Overproduction of free radicals manifests AFB_1_-induced neurotoxicity, dysregulation of lipid profile, glucose level, and insulin concentration, HOMA-IR, TNF-*α*, and IDO, increased activity of AChE and MAO, and inhibition of the antioxidant enzymes, HOMA-B, and TIMP3. These processes intensify oxidative stress. The factors used in this study did not have a significant effect on the urea concentration in brains of rats. Moreover, changes in histology of brain are visible after exposure to AFB_1_. ALE, a potent antioxidant, reduced free radical production and increased antioxidant enzyme activity. These ALE-mediated effects are significant in overcoming oxidative stress. Moreover, joint treatment using ALE and AFB_1_ alleviates the histopathological features induced by the exposure to AFB_1_. ALE can be successfully considered as a possible nominee for controlling neurotoxicity resulting from food and feed contaminated with AFB_1_, which causes numerous harmful effects on humans and animals' health. The phenolic compounds present in natural, balanced proportions in ALE have beneficial effects on the brain. The neuroprotective effect of ALE involves the regulation of lipid metabolism and the alleviation of inflammation and oxidative stress.

The article "Artichoke Leaf Extract-Mediated Neuroprotection against Effects of Aflatoxin in Male Rats" was published in 2022. Journal: Biomed Res Int.

## Figures and Tables

**Figure 1:** (a) HPLC chromatogram of aqueous extract of the artichoke (*Cynara scolymus* L.) leaf extract capsule and (b) list of the components of the artichoke capsule and their concentrations.

**Figure 2:** Mean ± SD of total lipids (a), cholesterol (b), triglycerides (c), HDL (d), LDL (e), and VLDL (f) in plasma of male rats treated with AFB1, ALE, and their combination for 42 days. Abbreviations: control: animals treated with water; DMSO: animals treated with DMSO (solvent); ALE: animals treated with artichoke leaves extract (100 mg/kg body weight); AFB1: animals treated with Aflatoxin B1 (72 *μ*g/kg body weight); ALE+AFB1: animals treated with a combination of artichoke extract and aflatoxin B1; LDL: low-density lipoprotein; VLDL: very low-density lipoprotein; HDL: high-density lipoprotein. The same letter (A, B, C, D, and E) denote no significant difference among experimental groups (*p* < 0.05; *n* = 5; LSD, ANOVA test).

**Figure 3:** Mean ± SD of glucose (a) and insulin (b) concentration, HOMA-IR (c), and HOMA-B (d) index in plasma of male rats treated with AFB1, ALE, and their combination for 42 days. Abbreviations: HOMA-IR: homeostatic model assessment for insulin resistance; HOMA-B: homeostatic model assessment for beta cells; for other explanations, see Figure 1.

**Figure 4:** Mean ± SD concentration of TNF*α* (a), IDO (b), and TIMP3 (c) in the brain of male rats treated with AFB1, ALE, and their combination for 42 days. Abbreviations: TNF*α*: tumor necrosis factors *α*; IDO: indoleamine-pyrrole 2,3-dioxygenase; TIMP3: tissue inhibitor metallopeptidase; for other explanations, see Figure 1.

**Figure 5:** Mean ± SD concentration of TBARS (a), activity of XO (b), and concentration of UA (c) in the brain of male rats treated with AFB1, ALE, and their combination for 42 days. Abbreviations: TBARS: thiobarbituric acid reactive substances; XO: xanthine oxidase; UA: uric acid; for other explanations, see Figure 1.

**Figure 6:** Mean ± SD concentration of GSH (a) and activity of SOD (b), GST (c), and GPx in the brain of male rats treated with AFB1, ALE, and their combination for 42 days. Abbreviations: GSH: glutathione reduced form; SOD: superoxide dismutase; GST: glutathione S-transferase; GPx: glutathione peroxidase; for other explanations, see Figure 1.

The article "Artichoke Leaf Extract-Mediated Neuroprotection against Effects of Aflatoxin in Male Rats" was published in 2022. Journal: Biomed Res Int.

**Figure 7:** Mean ± SD activity of AChE (a) and MAO (b) and concentration of NO (c) and urea (d) in the brain of male rats treated with AFB1, ALE, and their combination for 42 days. Abbreviations: AChE: acetylcholinesterase; MAO: monoamine oxidase; NO: nitric oxide; for other explanations, see Figure 1.

**Figure 8:** Principal component analysis (PCA) to evaluate similarities among all the parameters measured in the brain or plasma of male rats treated with AFB1 (aflatoxin B1-72 *μ*g/kg body weight), ALE (artichoke leaves extract -100 mg/kg body weight), and their combination for 42 days. (a) PCA analysis of variables. (b) PCA analysis of cases. Abbreviations: see Figures 1–6.

**Figure 9:** Representative H&E-stained brain samples of male rats from the control group, ALE group (artichoke leaves extract -100 mg/kg body weight), AFB1 group (aflatoxin B1 -72 *μ*g/kg body weight), and ALE+AFB1 group (artichoke leaves extract -100 mg/kg body weight+aflatoxin B1-72 *μ*g/kg body weight). Abbreviations: CA1, 2, 3: cornu ammonis 1, 2, 3; DG: dentate gyrus; Sp: stratum pyramidalis; Sr: stratum radiatum; So: stratum oriens; for other explanations, see Figure 1.

## Data Availability

All data related to the MS are provided in this work.
